# Schisandrin B Diet Inhibits Oxidative Stress to Reduce Ferroptosis and Lipid Peroxidation to Prevent Pirarubicin-Induced Hepatotoxicity

**DOI:** 10.1155/2022/5623555

**Published:** 2022-07-18

**Authors:** Hongwei Shi, Yue Yan, Hong Yang, Peng Pu, Heng Tang

**Affiliations:** ^1^Department of Radiation Oncology, Hubei Cancer Hospital, Tongji Medical College, Huazhong University of Science and Technology, Wuhan, China; ^2^Department of Oncology, Renmin Hospital of Wuhan University, Wuhan, China; ^3^College School of Traditional Chinese Medicine, Chongqing Medical University, Chongqing 400016, China; ^4^Department of Endocrine, The First Affiliated Hospital of Chongqing Medical University, Chongqing, China; ^5^Department of Cardiology, The First Affiliated Hospital of Chongqing Medical University, Chongqing, China; ^6^Department of Cardiology, Southwest Hospital, Third Military Medical University (Army Medical University), Chongqing 400038, China

## Abstract

**Objective:**

Pirarubicin (THP) is one of anthracycline anticancer drugs. It is widely used in the treatment of various cancers, but its hepatotoxicity cannot be ignored. Schisandrin B (SchB) is a traditional liver-protecting drug, which has the ability to promote mitochondrial function and upregulate cellular antioxidant defense mechanism. However, whether it can resist THP-induced hepatotoxicity has not been reported. The purpose of this study was to observe and explore the effect of SchB on THP-induced hepatotoxicity and its potential mechanism by adding SchB to the diet of rats with THP-induced hepatotoxicity.

**Methods:**

The rat model of THP-induced hepatotoxicity was established and partly treated with SchB diet. The changes of serum liver function indexes ALT and AST were observed. The histomorphological changes of liver were observed by HE staining. The biomarker levels of oxidative stress in rat serum and liver were measured to observe oxidative stress state. The expressions of ferroptosis-related protein GPX4 and oxidative stress-related protein were detected by Western blot. Primary hepatocytes were prepared and cocultured with THP, SchB, and Fer-1 to detect the production of reactive oxygen species (ROS) and verify the above signal pathways.

**Results:**

THP rats showed a series of THP-induced hepatotoxicity changes, such as liver function damage, oxidative stress, and ferroptosis. SchB diet effectively alleviated these adverse reactions. Further studies showed that SchB had strong antioxidant and antiferroptosis abilities in THP-induced hepatotoxicity.

**Conclusion:**

SchB has obvious protective effect on THP-induced hepatotoxicity. The mechanism may be closely related to inhibiting oxidative stress and ferroptosis in the liver.

## 1. Introduction

Pirarubicin (THP), the third generation of anthracycline antitumor drugs, has gradually replaced the first generation of anthracycline antitumor drugs represented by adriamycin in clinic because of its better antitumor effect and less toxic and side effects [1]. However, THP has strong toxic and side effects, which seriously affects its clinical application [2]. In cells, THP can induce the production of oxygen free radicals, trigger abnormal iron metabolism, apoptosis, calcium overload, and mitochondrial damage, and destroy the structure and function of cell membrane [3–5]. Relevant reports pointed out that in patients who died of chemotherapy drugs, diffuse hemosiderin, intracellular ferritin and serum iron concentration increased, and transferrin saturation could be as high as 87%, indicating that iron ions may play an important role in the toxic and side effects of THP [6]. THP leads to the increase of ROS production, resulting in the process of reactive oxygen species (ROS) oxidation biofilm in the process of lipid peroxidation and the decrease of the expression of antioxidant system (GSH and GPX4), which triggers ferroptosis [5, 7]. In addition, the accumulation of intracellular iron caused by ferroptosis leads to the increase of toxic lipid peroxide ROS, forming a vicious circle [7, 8]. Our previous studies have shown that THP can cause oxidative stress and apoptosis in cardiomyocytes. In addition, THP can also cause hepatotoxicity, which may be related to the metabolism of THP in the liver after entering the blood system. However, how THP causes hepatotoxicity is unknown.

Oxidative stress is an imbalance between the production and accumulation of ROS such as superoxide radical (O^2-^), hydrogen peroxide (H_2_O_2_), and hydroxyl radical (^−^OH) in cells and tissues and antioxidant factors in biological systems [9]. It is usually stimulated by radiation, pollution, heavy metals, and chemicals, which has a harmful impact on important cell structures such as proteins, lipids, and nucleic acids [9]. Malondialdehyde blood concentration is often used to evaluate lipid peroxidation and is also a useful marker of oxidative stress [10]. There is also an antioxidant defense system in cells and tissues, such as superoxide dismutase (SOD), catalase (CAT), and glutathione peroxidase (GPX), to protect themselves against ROS [9, 11]. There is a lot of evidence that oxidative stress plays a major role in several common diseases, including cancer, obesity, diabetes, metabolic disorders, liver diseases, atherosclerosis, and cardiovascular disease [9, 11, 12]. Oxidative stress also plays an important role in some other diseases, such as obstructive sleep apnea syndrome, ankylosing spondylitis, Alzheimer's disease, and Parkinson's disease [13–15].

Schisandrin B (SchB) is a traditional Chinese medicine monomer extracted from Schisandra chinensis (Turcz) Baillon, which widely exists in tonic prescriptions [16, 17]. It is a biphenyl cyclooctene lignan, which is especially commonly used in the treatment of liver diseases [16, 18]. Early studies have shown that SchB can protect many organs including the liver, heart, kidney, brain, and skin, especially the liver from toxic substances and free radical damage [18–20]. Relevant research also points out that SchB can protect mice from hepatotoxicity caused by various drugs [21–24]. Its hepatoprotective effect is related to the antioxidant and glutathione redox state [24]. Oxidative stress and glutathione antioxidant system are closely related to cell ferroptosis [25]. In addition, SchB can also improve liver mitochondria and hinder the membrane permeability conversion induced by calcium ions, so as to prevent apoptosis under high oxidative pressure [23]. These characteristics of SchB make it have the potential to develop into a first-class raw material for functional foods, herbal dietary supplements, antiaging health care products, and skin care products. As a way of dietotherapy, SchB has the potential to protect tissues from oxidative damage caused by drug damage, environmental harmful substances, strenuous exercise, aging, and other factors. However, it is unknown whether SchB can protect the liver from THP injury.

In this study, we explored the role of SchB in THP-induced hepatotoxicity in vivo and in vitro. For its mechanism, we explored the role of oxidative stress and ferroptosis in THP-induced hepatotoxicity and the therapeutic effect of SchB.

## 2. Materials and Methods

### 2.1. Materials

SchB and THP were purchased from Shanghai Aladdin Reagent Co., Ltd. (Shanghai, China). Ferrostatin-1 (Fer-1) was purchased from MedChemExpress. Commercial kits for measuring alanine aminotransferase (ALT), aspartate aminotransferase (AST), malondialdehyde (MDA, A003-1-2), superoxide disproportionation (SOD, A001-3-2), glutathione (GSH, A006-2-1), glutathione peroxidase (GSH-px, A005-1-2), catalase (CAT, A007-1-1), and total antioxidant capacity (T-AOC, A015-1-2) were purchased from Nanjing Jiancheng Bioengineering Institute. Iron assay kit (ab83366) was purchased from Abcam. ROS detection kit (BL714A) and CCK-8 cell viability and toxicity detection kit (BS350B) were derived from Biosharp (Anhui, China). Antibodies recognizing nuclear factor erythroid 2 like 2 (NRF2, Cat No. 16396-1-AP), NADPH oxidase 2/4 (NOX2/4, Cat No. 19013-1-AP/14347-1-AP), superoxide disproportionation 2 (SOD2, Cat No. 24127-1-AP), glutathione peroxidase 4 (GPX4, Cat No. 14432-1-AP), B-cell lymphoma-2 (Bcl-2, Cat No. 12789-1-AP), Bcl-2-associated X (Bax, Cat No. 50599-2-Ig), and glyceraldehyde-3-phosphate dehydrogenase (GAPDH, Cat No. 10494-1-AP) were bought from Proteintech (Wuhan, China). All other chemicals and reagents were analytical grade.

### 2.2. Animal Studies

#### 2.2.1. Animal Model and Diet

Studies were approved by the Animal Care Use Committee of the First Affiliated Hospital of Chongqing Medical University (CMU). SD rats were maintained in accordance with the guidelines published by the US National Institutes of Health (NIH). This study was conducted in compliance with the Guide for the Care and Use of Laboratory Animals published by the National Academy Press (NIH). During the animal experiment, the investigator was blinded to the group allocation. A total of 40 male SD rats (180~200 g, 6~8 weeks) were purchased from the CMU experimental animal center.

The rats were randomly divided into four groups: control (CON) group (normal diet rats were injected with equal volume of normal saline through caudal vein once a week, *n* = 10), SchB group (SchB diet rats, 50 mg/kg/day, were injected with equal volume of normal saline through caudal vein once a week, *n* = 10), THP group (normal diet rats were injected with 3 mg/kg/day THP through caudal vein once a week, *n* = 10), and SchB+THP group (SchB diet rats, 50 mg/kg/day, were injected with 3 mg/kg/day THP through caudal vein once a week, *n* = 10). CON and THP rats were fed an AIN-76A feed (12.4% fat, 68.8% carbohydrate, and 18.8% protein). SchB and SchB+THP rats were fed an SchB feed (approximately 0.5‰ SchB was added into AIN-76A feed). After conversion, 0.5‰ SchB in feed = 50 mg/kg in rats. AIN-76A feed and the processing of SchB feed was completed by Jiangsu Synergy Pharmaceutical Bioengineering Co., Ltd. The survival of rats was recorded every day, and the food consumption and body weight were recorded twice a week.

Similar feed processing, feeding schemes, and the dose of THP and SchB could be found in our previous studies [19, 26, 27].

#### 2.2.2. Sample Collection and Preparation

At study end, overnight fasted animals were sacrificed by cervical dislocation after body weight was measured under anesthesia (inhalation of 2% isoflurane). Rat blood samples were obtained from the abdominal aorta. To isolate serum, blood samples were collected and centrifuged at 3000 rpm for 30 min at 4°C. The livers were also removed and measured. A part of the livers was used for histological analysis, and the remaining livers were used for molecular analyses. Liver/body weight (mg/g) = liver weight (mg)/body weight (g).

#### 2.2.3. Biochemical Analysis

ALT, AST, MDA, SOD, GSH, GSH-px, CAT, and T-AOC levels in serum were assayed according to the kit protocols. A proper amount of liver tissue was homogenized in normal saline at a ratio of 1 : 10 and then centrifuged in a low-temperature centrifuge at 12000 rpm for 15 minutes. The supernatant was obtained to determine the content of MDA, SOD, GSH, GSH-px, CAT, and T-AOC. The contents of total iron, Fe^2+^, and Fe^3+^ in the liver were measured according to iron assay kit test instructions. Fe^3+^ = total iron (Fe^2+^ + Fe^3+^) − Fe^2+^.

#### 2.2.4. Histological Analysis

Liver tissues were excised, washed in saline solution, and fixed in 10% formalin. Several tissue sections (thickness = 4 ~ 5 *μ*m) were prepared and stained in hematoxylin and eosin (H&E) for histopathology. Staining images were observed with Nikon eclipse 80i microscope (Nikon, Chiyoda, Japan) at 200x magnification.

### 2.3. Cell Experiments

#### 2.3.1. Cell Culture

Primary hepatocyte cultures were prepared as described in the previous studies. The cells were seeded at 8 × 10^5^ cells/well in 60 mm culture plates containing Dulbecco's Modified Eagle Medium/Nutrient Mixture F-12 (DMEM/F12) medium supplemented (Gibco, China) with 10% fetal bovine serum (Pan, Germany) and penicillin/streptomycin (Beyotime Biotechnology, China). After 48 h, the culture medium was replaced every two days.

#### 2.3.2. CCK-8 Kit Was Used to Determine the Optimal Concentration of THP and the Coculture Effect of THP and SchB

We used CCK-8 cell viability test kit to explore the optimal concentration of THP and SchB on hepatocyte. Hepatocyte was treated with 0, 2.5, 5, 10, and 20 *μ*M THP for 6, 12, 24, and 48 h to establish hepatocyte injury model. The concentration of SchB treatment was divided into 25 *μ*M, 50 *μ*M, 100 *μ*M, and 200 *μ*M and cocultured with the optimal concentration of THP to detect cell viability. The cell viability of CON was defined as 100%.

#### 2.3.3. Hepatocyte Grouping and Treatment

For experiments, primary hepatocytes were pretreated with 50 *μ*M SchB (dissolved in DMSO) or 5 *μ*M Fer-1 (dissolved in DMSO) or equivalent DMSO for 2 h and then incubated with 5 *μ*M THP (dissolved in DMSO) or equivalent DMSO for 24 h. In short, hepatocytes were divided into 6 groups: CON group (equivalent DMSO, 26 h), SchB group (50 *μ*M, 26 h), Fer-1 group (5 *μ*M, 26 h), THP group (equivalent DMSO, 2 h; then 5 *μ*M THP, 24 h), SchB+THP group (50 *μ*M SchB, 2 h; then 50 *μ*M SchB+5 *μ*M THP, 24 h), and Fer-1+THP group (5 *μ*M Fer-1, 2 h; then 5 *μ*M Fer-1+5 *μ*M THP, 24 h).

#### 2.3.4. ROS Staining in Hepatocyte

Hepatocyte was seeded into 24-well plates and treated according to the cell treatment scheme mentioned above. When the cell growth reached 70%-80%, the staining was carried out according to the instructions of ROS staining kit. Then, the positive area was counted by ImageJ software (ImageJ 1.51J8).

### 2.4. Western Blotting

For Western blotting, liver tissues and primary hepatocytes were lysed in radioimmunoprecipitation (RIPA) lysis buffer (Beyotime Biotechnology) with 1% protease inhibitor (Beyotime Biotechnology) in 4°C for 30 min. Supernatants were collected after centrifuging in 4°C at 12000 rpm for 15 minutes, and protein concentrations were determined using a bicinchoninic acid assay (BCA) kit (Beyotime Biotechnology). Add 1/4 volume of 5x protein loading buffer (Beyotime Biotechnology) to the supernatant, and then, heat it to 100°C for 10 min to denature the protein. In total, about 50 *μ*g heart tissue lysate or 20 *μ*g cell lysate was used for 12% sodium dodecyl sulfate-polyacrylamide gel electrophoresis (SDS-PAGE), and proteins were then transferred to an FL membrane (Millipore) at 4°C for 1.5 h. After blocking with 5% nonfat milk powder (Beyotime Biotechnology) at room temperature for 1.5 h, the following primary antibodies were added and incubated overnight at 4°C: NRF2 (1 : 1000), NOX2/4 (1 : 1000), GPX4 (1 : 1000), SOD2 (1 : 1000), cleaved caspase-3 (1 : 1,000), Bax (1 : 1000), and Bcl-2 (1 : 1000). Subsequently, HRP-conjugated goat anti-rabbit IgG (H+L) secondary antibodies (1 : 10000; Thermo Fisher Scientific, Inc.; cat. no. 31460) were added and incubated at room temperature for 1.5 h. The Western blotting results were analyzed using BeyoECL Plus (Beyotime Institute of Biotechnology) and Image Lab software (version 5.2.1; Bio-Rad Laboratories, Inc.). The specific protein expression levels were normalized to that of GAPDH.

### 2.5. Statistical Analysis

Data were expressed as the mean ± standard error of the mean (SEM). The normal distribution and variance homogeneity of the data are detected, and then, the significant differences between groups were statistically analyzed using a one- or two-way analysis of variance, followed by Tukey's multiple-comparison post hoc test. *P* values ≤ 0.05 were considered statistically significant.

## 3. Results

### 3.1. SchB Diet Significantly Increased Body Weight and Feed Consumption in THP-Induced Hepatotoxicity Rats

From the third week of the study, THP rats gained lower body weight than CON rats (Figure 1(a)). At the same time, SchB diet significantly increased the weight loss (Figure 1(a)). From the fourth week, these differences were more significant. Similarly, THP also reduced feed consumption compared to CON rats, and SchB diet significantly increased the feed consumption (Figure 1(b)).

### 3.2. SchB Diet Significantly Decreased Death Rate and Liver/Body Weight of THP-Induced Hepatotoxicity Rats

The establishment of the whole animal model lasted for 56 days (8 weeks). In THP group, five of the 10 rats died (died on days 38, 43, 44, 48, and 53, respectively), with a mortality rate of 50% (Figure 1(c)). In SchB+THP group, one of the 10 rats died (died on day 54), with a mortality rate of 10% (Figure 1(c)). In CON and SchB groups, no rats died (Figure 1(c)). On the other hand, the liver/body weight increased in THP rats but decreased after feeding SchB diet (Figure 1(d)).

### 3.3. The Effects of SchB Diet on Serum Biochemical Indexes of THP-Induced Hepatotoxicity Rats

The levels of ALT (Figure 2(a)) and AST (Figure 2(b)) increased in serum of THP rats, which indicated that THP caused hepatotoxicity in rats. Similarly, the serum biochemical indexes of oxidative stress in rats were also abnormal, such as the increase of MDA (Figure 2(c)) and the decrease of SOD (Figure 2(d)), GSH (Figure 2(e)), GSH-px (Figure 2(f)), CAT (Figure 2(g)), and 2T-AOC (Figure 2(h)). It is a wonder that all the abnormal serum biochemical indexes were reversed after feeding SchB diet.

### 3.4. Effect of SchB Diet on Hepatic Histology Liver Biochemical Indexes of THP-Induced Hepatotoxicity Rats

H&E staining (Figure 3(a)) revealed that the liver in the CON rats showed normal architecture, and apparent injuries were found in THP rats, such as granular and vacuolar degeneration, macro- and microvesicular steatosis, parenchymal mononuclear cell infiltration, and pyknotic nuclei in hepatocytes, which were all restored by feeding SchB diet. Similarly, the liver biochemical indexes of oxidative stress in rats were also abnormal, such as the increase of MDA (Figure 3(b)) and the decrease of SOD (Figure 3(c)), GSH (Figure 3(d)), GSH-px (Figure 3(e)), CAT (Figure 3(f)), and 3T-AOC (Figure 3(g)). It is a wonder that all the abnormal liver biochemical indexes were reversed after feeding SchB diet.

### 3.5. SchB Diet Inhibited Ferroptosis and Oxidative Stress on the Liver of THP-Induced Hepatotoxicity Rats

The contents of total Fe (Figure 4(a)), Fe^2+^ (Figure 4(b)), and Fe^3+^ (Figure 4(c)) in the liver of THP rats increased, which also decreased after feeding SchB diet.

As shown in Figure 4(d), the expression of NRF2, GPX4, SOD2, and Bcl-2/Bax decreased, while the expression of NOX2/4 and cleaved caspase-3 increased in the liver of THP rats. However, the above changes were significantly reversed after feeding SchB diet. Semiquantitative analysis provides more evidence (Figure 4(e)).

### 3.6. The Optimal Concentration of THP and SchB on Hepatocytes

As shown in Figure 5(a), we detected the effect of four concentrations of THP on cell activity after 24 h treatment. The results showed that when THP concentration was 2.5 *μ*M, it had little effect on cell viability, and there was no significant difference compared with CON. When THP concentrations were 10 and 20 *μ*M, the cell viability decreased too sharply and the cell mortality was too high, which was not suitable for cell research. Therefore, 5 *μ*M THP concentration was selected for subsequent cell experiments.

As shown in Figure 5(b), under the condition of 50 *μ*M THP-induced cell injury, we detected the effects of four concentrations of SchB on cell viability. Although the cell viability of 25 *μ*M SchB-treated cells increased slightly, there was no difference compared with THP group. 50 *μ*M, 100 *μ*M, and 200 *μ*M concentrations of SchB treatment of hepatocytes significantly improved the decreased cell viability, but there was no difference among the three groups. Therefore, SchB concentration of 50 *μ*M was selected for subsequent cell experiments.

### 3.7. SchB Inhibited Ferroptosis and Oxidative Stress on Hepatocytes Cultured with THP

As shown in Figure 5(c), THP induced hepatocytes to produce a large amount of ROS, which decreased after both SchB and Fer-1 treatment. ROS was almost absent in CON, SchB, and Fer-1 groups. The relative fluorescence intensity provides more evidence (Figure 5(d)).

As shown in Figure 5(e), the expression of NRF2, GPX4, SOD2, and Bcl-2/Bax decreased, while the expression of NOX2/4 and cleaved caspase-3 increased in THP hepatocytes. However, the above changes were significantly reversed after SchB or Fer-1 treatment. Semiquantitative analysis provides more evidence (Figure 5(f)).

## 4. Discussion

Our study found that THP led to the decrease of body weight and food intake of rats, and the general state was poor. In addition, THP rats showed an increase in the liver/body weight. In normal, the ratio of liver to body weight is relatively constant, but after the animals were poisoned, the liver coefficient increased, indicating that the functions of organs such as congestion, edema or hyperplasia, and hypertrophy decreased [28]. In the group of rats treated with pirarubicin alone, the mortality rate of rats is higher, up to 40%. There are also cases of poor quality of life and even death caused by pirarubicin and its family drugs in clinic, but the mortality rate is not high [29]. The specific reason may be that the clinical medication interval is usually more than 1 month, the cumulative dose of drug organotoxicity is often more than 6 months, and the medication methods are slightly different (such as slow drip administration) [30]. In animal studies, the drug interval is 1 week, the time to reach the accumulated dose is 2 months, and it is direct caudal vein injection, which may be more toxic. And the clinical medication plan is safer, which can monitor the general situation and organ function of patients, change the drug plan, and reduce or stop the drug at any time [30, 31].

Our study also found that THP can also cause hepatotoxicity in rats, resulting in abnormal increase of biochemical markers related to hepatotoxicity, such as ALT and AST. In order to find out how THP causes hepatotoxicity, we detected the biochemical markers related to oxidative stress in serum and liver tissue. The results showed that the levels of SOD, GSH, GSH-px, CAT, and T-AOC decreased abnormally, while MDA increased abnormally, indicating that THP led to abnormal oxidative stress in rat liver. SOD is considered to be the main destruction factor of oxygen free radicals in vivo, which can resist the cell damage caused by oxygen free radicals and repair the damaged cells [32, 33]. In addition, the decreased levels of GSH, GSH-px, CAT, and T-AOC are also considered to have abnormal oxidative stress in cell [32–35]. MDA is considered to be one of the final products of oxidation reaction, which leads to the cross-linking and polymerization of many key macromolecules, such as protein and nucleic acid, which induces cytotoxicity and affects organ function [32, 33]. NOX2/4 are two important NADPH oxidase and the main sources of reactive oxygen species [36, 37]. The increased expression of NOX2/4 in rat liver also showed that THP induced ROS overproduction. Excessive ROS will oxidize the biofilm, which can lead to lipid peroxidation and damage the cell membrane, so as to change the fluidity and permeability of the cell membrane and finally lead to the change of cell structure and function [38, 39]. Lipid peroxidation is closely related to ferroptosis [7, 39]. Fe^2+^ can catalyze the highly expressed unsaturated fatty acids on the cell membrane to produce lipid peroxidation [40]. The iron-dependent accumulation of lipid peroxidation can induce ferroptosis after reaching the lethal level [7]. On the other hand, depletion of intracellular GSH will lead to inactivation of GPX4 and accumulation of lipid peroxidation, which can also induce cell death to a certain extent [41–43]. Consistent with our results, the expression of GPX4 decreased in the liver of THP rats, while total iron ion, Fe^2+^, and Fe^3+^ increased, indicating that THP eventually led to lipid peroxidation and ferroptosis in the liver of rats. Relevant studies have also pointed out that excessive ROS will also induce apoptosis by activating caspase family proteins and Bcl-2/Bax [44]. In our study, the expression of cleaved caspase-3 increased and the expression of Bcl-2/Bax decreased, indicating that THP also induced liver cell apoptosis in addition to lipid peroxidation and ferroptosis.

T. Fedotcheva and N. Fedotcheva's study pointed out that adriamycin can act on mitochondrial permeability transition pore (mPTP) and respiratory complex II, causing ferroptosis of liver and cardiomyocytes, that is, iron-dependent cell death driven by membrane injury [45]. In our previous studies, the abnormal opening of mPTP led to the release of cytochrome c from mitochondria and activated caspase apoptosis pathway, and mPTP is often considered to be one of the key factors leading to apoptosis [19]. Surprisingly, mPTP may also cause ferroptosis, which may also be the key factor leading to hepatocyte apoptosis and ferroptosis in this study, but further research is needed to prove it. Yu et al. showed that high-iron diet can lead to ferroptosis in hepatocytes, eventually leading to liver fibrosis and impaired function; CCl4, a classical hepatotoxic chemical, can also cause liver damage by ferroptosis; the levels of serum transferrin and liver transferrin in clinical patients with liver cirrhosis are significantly reduced, and the levels of liver iron and lipid peroxidation are also significantly increased [46]. These evidences suggest that ferroptosis may be a common potential therapeutic target for hepatotoxicity caused by various causes.

Another important finding is that SchB has a good protective effect on THP-induced hepatotoxicity. Our previous studies have shown that SchB can improve THP-induced cardiotoxicity in rats through antioxidant stress characteristics [19, 26]. Relevant studies have also shown that SchB can stimulate the protective response of hepatocytes in experimental rats, improve the oxidation state of liver, and reduce the hepatotoxicity of mercury dichloride and carbon tetrachloride [24, 47]. In this study, SchB also increased the levels of SOD, GSH, GSH-px, CAT, and T-AOC, decreased the level of MDA, and inhibited the abnormal oxidative stress in the liver. Similarly, lipid peroxidation, ferroptosis, and apoptosis caused by oxidative stress were also inhibited.

It is worth noting that in our in vitro study, Fer-1 inhibited ferroptosis and lipid peroxidation, as well as apoptosis. Fer-1, a selective ferroptosis inhibitor and synthetic antioxidant, prevents the damage of membrane lipids through the reduction mechanism, so as to inhibit cell death [5, 46]. Since ferroptosis is an iron dependent and new programmed cell death mode different from apoptosis, cell necrosis, and autophagy, we speculate that the effect of Fer-1 on inhibiting apoptosis may be to reduce ROS in liver cells and inhibit apoptosis through its antioxidant properties [48–51].

Our study confirmed that the liver protective effect of SchB as a natural molecule depends on reducing the level of oxidative stress, thereby inhibiting lipid peroxidation, ferroptosis, and apoptosis. However, the specific mechanism of SchB-regulating oxidative stress, ferroptosis, and apoptosis in vivo is not completely clear. Therefore, further research is needed to clarify the potential role of SchB as a new and effective antioxidant, antiferroptosis, and antiapoptotic drug in drug-induced liver diseases and even other liver diseases.

## 5. Conclusion

Although cardiotoxicity is the main side effect of THP, its hepatotoxicity cannot be ignored, which also sounded an alarm for cancer treatment. As a dietary additive, SchB has outstanding potential in the prevention and treatment of THP-induced hepatotoxicity model and hepatocyte injury model in rats. The mechanism may be related to inhibiting oxidative stress to reduce ferroptosis and lipid peroxidation. This study clarified the mechanism of SchB in THP-induced hepatotoxicity and provided a theoretical basis for the use of SchB as a dietary therapy scheme combined with clinical drugs in the future.

## 6. Limitations

Although this study proves the potential role of ferroptosis in the prevention and treatment of THP-induced hepatotoxicity by SchB to a certain extent, there are still some limitations. For example, how SchB and THP affect GPX4-mediated ferroptosis (specific molecular mechanism) is not clear and not verified in GPX4 knockout and overexpression animals; the key role of mPTP in hepatocyte apoptosis and ferroptosis is not clear. These problems are also the next research plan of the research group, which needs further research and exploration.

## Figures and Tables

**Figure 1:** The effect of SchB diet on the body weight, feed consumption, survival, and liver/body weight in THP-induced hepatotoxicity rats. From the third week, THP rats gained lower body weight (a) and feed consumption (b) than CON rats. At the same time, SchB diet could significantly improve the body weight (a) of THP rats. From the fourth week, the feed consumption (b) was significantly improved by SchB diet in THP rats. At the end of eighth week, there is no death in CON and SchB diet rats (c). But in THP, the death rate was 50%, and after SchB diet, the death rate rise to 90% (c). The THP rats also gained liver/body weight increased compared with CON rats, and SchB diet significantly decreased liver/body weight in THP rats (d). Values are expressed as mean ± SEM. ^∗^*P* < 0.05, ^∗∗^*P* < 0.01, and ^∗∗∗∗^*P* < 0.0001 THP vs. CON; ^#^*P* < 0.05, ^##^*P* < 0.01, and ^####^*P* < 0.0001 SchB+THP vs. THP. CON: control; SchB: schisandrin B; THP: pirarubicin.

**Figure 2:** Effects of SchB diet on serum biochemical indices in THP-induced hepatotoxicity rats. THP induced the increase of ALT (a), AST (b), and MDA (c) and the decrease of SOD (d), GSH (e), GSH-px (f), CAT (g), and T-AOC (h) in serum of rats, while in the THP rats with SchB diet, these abnormal indexes were reversed (a–h). Values are expressed as mean ± SEM. ^∗^*P* < 0.05 vs. CON and ^#^*P* < 0.05 vs. THP. CON: control; SchB: schisandrin B; THP: pirarubicin; ALT: alanine aminotransferase; AST: aspartate aminotransferase; MDA: malondialdehyde; SOD: superoxide disproportionation; GSH: glutathione; GSH-px: glutathione peroxidase; CAT: catalase; T-AOC: total antioxidant capacity.

**Figure 3:** Effect of SchB diet on liver of THP-induced hepatotoxicity rats. The effect of SchB and THP in hepatic histology (a). THP induced the increase of MDA (b) and the decrease of SOD (c), GSH (d), GSH-px (e), CAT (f), and T-AOC (g) in the liver of rats, while in the THP rats with SchB diet, these abnormal indexes were reversed (c–g). Values are expressed as mean ± SEM. ^∗^*P* < 0.05 vs. CON and ^#^*P* < 0.05 vs. THP. CON: control; SchB: schisandrin B; THP: pirarubicin; NS: normal saline; MDA: malondialdehyde; SOD: superoxide disproportionation; GSH: glutathione; GSH-px: glutathione peroxidase; CAT: catalase, T-AOC: total antioxidant capacity.

**Figure 4:** SchB diet inhibited ferroptosis and oxidative stress on liver of THP-induced hepatotoxicity rats. The levels of total Fe (a), Fe^2+^ (b), and Fe^3+^(c) decreased in the liver of THP rats. The levels of NRF2, SOD2, GPX4, and Bcl-2/Bax decreased in the liver of THP rats (d). In addition, the expression of NOX2/4 and cleaved caspase-3 was slightly increased (d). However, SchB diet eliminated these adverse reactions (a–d). Semiquantitative analysis provides more evidence (e). Values are expressed as mean ± SEM. ^∗^*P* < 0.05 vs. CON and ^#^*P* < 0.05 vs. THP. CON: control; SchB: schisandrin B; THP: pirarubicin; NRF2: nuclear factor erythroid 2 like 2; NOX2/4: NADPH oxidase 2/4; SOD2: superoxide disproportionation 2; GPX4: glutathione peroxidase 4; Bcl-2: B-cell lymphoma-2; Bax: Bcl-2-associated X.

**Figure 5:** SchB inhibited ferroptosis and oxidative stress on hepatocytes cultured with THP. Effects of different concentrations of THP on cell viability (a). Effects of different concentrations of SchB with 5 *μ*M THP on cell viability (b). The levels of ROS increased, which decreased with Fer-1 or SchB treatment in THP hepatocytes (c). The relative fluorescence intensity provides more evidence (d). The levels of NRF2, SOD2, GPX4, and Bcl-2/Bax decreased in THP hepatocytes (e). In addition, the expression of NOX2/4 and cleaved caspase-3 was slightly increased (e). However, SchB treatment eliminated these adverse reactions (e). Semiquantitative analysis provides more evidence (f). Values are expressed as mean ± SEM. ^∗^*P* < 0.05 vs. CON and ^#^*P* < 0.05 and ^&^*P* < 0.05 vs. THP. CON: control; SchB: schisandrin B; THP: pirarubicin; Fer-1: ferrostatin-1; NRF2: nuclear factor erythroid 2 like 2; NOX2/4: NADPH oxidase 2/4; SOD2: superoxide disproportionation 2; GPX4: glutathione peroxidase 4; Bcl-2: B-cell lymphoma-2; Bax: Bcl-2-associated X.

## Data Availability

The data used to support the findings of this study are available from the corresponding author upon request.

## References

[1] Mizutani H., Hotta S., Nishimoto A. (2017). Pirarubicin, an anthracycline anticancer agent, induces apoptosis through generation of hydrogen peroxide. *Anticancer Research*.

[2] Zhou J., Zhang X., Li M. (2013). Novel lipid hybrid albumin nanoparticle greatly lowered toxicity of pirarubicin. *Molecular Pharmaceutics*.

[3] Li Q., Qin M., Li T. (2020). Rutin protects against pirarubicin-induced cardiotoxicity by adjusting microRNA-125b-1-3p-mediated JunD signaling pathway. *Molecular and Cellular Biochemistry*.

[4] Li Q., Qin M., Tan Q. (2020). MicroRNA-129-1-3p protects cardiomyocytes from pirarubicin-induced apoptosis by down-regulating the GRIN2D-mediated Ca (2+) signalling pathway. *Journal of Cellular And Molecular Medicine*.

[5] Fang X., Wang H., Han D. (2019). Ferroptosis as a target for protection against cardiomyopathy. *Proceedings of the National Academy of Sciences of the United States of America*.

[6] Paglia D. E., Radcliffe R. W. (2000). Anthracycline cardiotoxicity in a black rhinoceros (Diceros bicornis): evidence for impaired antioxidant capacity compounded by iron overload. *Veterinary Pathology*.

[7] Yang W. S., Stockwell B. R. (2016). Ferroptosis: death by lipid peroxidation. *Trends In Cell Biology*.

[8] Su L. J., Zhang J. H., Gomez H. (2019). Reactive oxygen species-induced lipid peroxidation in apoptosis, autophagy, and ferroptosis. *Oxidative Medicine And Cellular Longevity*.

[9] Pizzino G., Irrera N., Cucinotta M. (2017). Oxidative stress: harms and benefits for human health. *Oxidative Medicine and Cellular Longevity*.

[10] Tsikas D. (2017). Assessment of lipid peroxidation by measuring malondialdehyde (MDA) and relatives in biological samples: analytical and biological challenges. *Analytical Biochemistry*.

[11] Jakubiak G. K., Osadnik K., Lejawa M., Kasperczyk S., Osadnik T., Pawlas N. (2021). Oxidative stress in association with metabolic health and obesity in young adults. *Oxidative Medicine and Cellular Longevity*.

[12] Jakubiak G. K., Osadnik K., Lejawa M. (2022). "Obesity and Insulin Resistance" Is the Component of the Metabolic Syndrome Most Strongly Associated with Oxidative Stress. *Antioxidants*.

[13] Stanek A., Brożyna-Tkaczyk K., Myśliński W. (2021). Oxidative stress markers among obstructive sleep apnea patients. *Oxidative Medicine and Cellular Longevity*.

[14] Stanek A., Cholewka A., Wielkoszyński T., Romuk E., Sieroń A. (2018). Decreased oxidative stress in male patients with active phase ankylosing spondylitis who underwent whole-body cryotherapy in closed cryochamber. *Oxidative Medicine and Cellular Longevity*.

[15] Kim G. H., Kim J. E., Rhie S. J., Yoon S. (2015). The role of oxidative stress in neurodegenerative diseases. *Experimental Neurobiology*.

[16] Nasser M. I., Zhu S., Chen C., Zhao M., Huang H., Zhu P. (2020). A comprehensive review on schisandrin B and its biological properties. *Oxidative Medicine and Cellular Longevity*.

[17] Liu C., Zhang S., Wu H. (2009). Non-thermal extraction of effective ingredients from Schisandra chinensis Baill and the antioxidant activity of its extract. *Natural Product Research*.

[18] Leong P. K., Ko K. M. (2016). Schisandrin B: a double-edged sword in nonalcoholic fatty liver disease. *Oxidative Medicine and Cellular Longevity*.

[19] Shi H., Tang H., Ai W. (2021). Schisandrin B antagonizes cardiotoxicity induced by Pirarubicin by inhibiting mitochondrial permeability transition pore (mPTP) opening and decreasing cardiomyocyte apoptosis. *Frontiers in Pharmacology*.

[20] Mou Z., Feng Z., Xu Z. (2019). Schisandrin B alleviates diabetic nephropathy through suppressing excessive inflammation and oxidative stress. *Biochemical and Biophysical Research Communications*.

[21] Ip S. P., Ko K. M. (1996). The crucial antioxidant action of schisandrin B in protecting against carbon tetrachloride hepatotoxicity in mice: a comparative study with butylated hydroxytoluene. *Biochemical Pharmacology*.

[22] Li Y. Z., Ma Z. N., Sun Y. S. (2018). Protective effects of extracts of Schisandra chinensis stems against acetaminophen-induced hepatotoxicity via regulation of MAPK and caspase-3 signaling pathways. *Chinese Journal Of Natural Medicines*.

[23] Chiu P. Y., Leung H. Y., Siu A. H., Poon M. K., Ko K. M. (2007). Schisandrin B decreases the sensitivity of mitochondria to calcium ion-induced permeability transition and protects against carbon tetrachloride toxicity in mouse livers. *Biological & Pharmaceutical Bulletin*.

[24] Deng Y., Xu Z., Xu B., Liu W., Feng S., Yang T. (2014). Antioxidative effects of schidandrin B and green tea polyphenols against mercuric chloride-induced hepatotoxicity in rats. *Journal of Environmental Pathology, Toxicology and Oncology*.

[25] Zhang Z., Guo M., Li Y. (2020). RNA-binding protein ZFP36/TTP protects against ferroptosis by regulating autophagy signaling pathway in hepatic stellate cells. *Autophagy*.

[26] Tang H., Zhao J., Feng R., Pu P., Wen L. (2022). Reducing oxidative stress may be important for treating pirarubicin-induced cardiotoxicity with schisandrin B. *Experimental and Therapeutic Medicine*.

[27] Shi H., Zeng Q., Wei Y. (2021). Canagliflozin is a potential cardioprotective drug but exerts no significant effects on pirarubicin-induced cardiotoxicity in rats. *Molecular Medicine Reports*.

[28] Zhang R., Zhang L., Jiang D. (2014). Mouse organ coefficient and abnormal sperm rate analysis with exposure to tap water and source water in Nanjing reach of Yangtze River. *Ecotoxicology*.

[29] Rawat P. S., Jaiswal A., Khurana A., Bhatti J. S., Navik U. (2021). Doxorubicin-induced cardiotoxicity: an update on the molecular mechanism and novel therapeutic strategies for effective management. *Biomedicine & Pharmacotherapy = Biomedecine & Pharmacotherapie*.

[30] Vejpongsa P., Yeh E. T. (2014). Prevention of anthracycline-induced cardiotoxicity: challenges and opportunities. *Journal of the American College of Cardiology*.

[31] Armenian S., Bhatia S. (2018). Predicting and preventing anthracycline-related cardiotoxicity. *American Society of Clinical Oncology Educational Book*.

[32] Yang W., Yuan W., Peng X. (2019). PPAR *γ*/Nnat/NF-*κ*B Axis involved in promoting effects of adiponectin on preadipocyte differentiation. *Mediators of Inflammation*.

[33] Zhang X., Xiong W., Chen L. L., Huang J. Q., Lei X. G. (2020). Selenoprotein V protects against endoplasmic reticulum stress and oxidative injury induced by pro-oxidants. *Free Radical Biology & Medicine*.

[34] Moretti E., Micheli L., Noto D., Fiaschi A. I., Menchiari A., Cerretani D. (2019). Resistin in human seminal plasma: relationship with lipid peroxidation, CAT activity, GSH/GSSG ratio, and semen parameters. *Oxidative Medicine And Cellular Longevity*.

[35] Pang Y. W., Jiang X. L., Wang Y. C. (2019). Melatonin protects against paraquat-induced damage during in vitro maturation of bovine oocytes. *Journal of Pineal Research*.

[36] Bedard K., Krause K. H. (2007). The NOX family of ROS-generating NADPH oxidases: physiology and pathophysiology. *Physiological Reviews*.

[37] Rezende F., Löwe O., Helfinger V. (2016). Unchanged NADPH oxidase activity in Nox1-Nox2-Nox4 triple knockout mice: what do NADPH-stimulated chemiluminescence assays really detect?. *Antioxidants & Redox Signaling*.

[38] Liu L., Zhang K., Sandoval H. (2015). Glial lipid droplets and ROS induced by mitochondrial defects promote neurodegeneration. *Cell*.

[39] Protchenko O., Baratz E., Jadhav S. (2021). Iron chaperone poly rC binding protein 1 protects mouse liver from lipid peroxidation and steatosis. *Hepatology*.

[40] Li N., Wang W., Zhou H. (2020). Ferritinophagy-mediated ferroptosis is involved in sepsis-induced cardiac injury. *Free Radical Biology & Medicine*.

[41] Chen X., Li J., Kang R., Klionsky D. J., Tang D. (2021). Ferroptosis: machinery and regulation. *Autophagy*.

[42] Qin X., Zhang J., Wang B. (2021). Ferritinophagy is involved in the zinc oxide nanoparticles-induced ferroptosis of vascular endothelial cells. *Autophagy*.

[43] Jelinek A., Heyder L., Daude M. (2018). Mitochondrial rescue prevents glutathione peroxidase-dependent ferroptosis. *Free Radical Biology & Medicine*.

[44] Saleh H., El-Shorbagy H. M. (2020). Chitosan protects liver against ischemia-reperfusion injury via regulating Bcl-2/Bax, TNF-*α* and TGF-*β* expression. *International Journal of Biological Macromolecules*.

[45] Fedotcheva T. A., Fedotcheva N. I. (2021). Protectors of the mitochondrial permeability transition pore activated by iron and doxorubicin. *Current Cancer Drug Targets*.

[46] Yu Y., Jiang L., Wang H. (2020). Hepatic transferrin plays a role in systemic iron homeostasis and liver ferroptosis. *Blood*.

[47] Xie Y., Hao H., Wang H., Guo C., Kang A., Wang G. (2014). Reversing effects of lignans on CCl_4_-induced hepatic CYP450 down regulation by attenuating oxidative stress. *Journal of Ethnopharmacology*.

[48] Miotto G., Rossetto M., Di Paolo M. L. (2020). Insight into the mechanism of ferroptosis inhibition by ferrostatin-1. *Redox Biology*.

[49] Kajarabille N., Latunde-Dada G. O. (2019). Programmed cell-death by Ferroptosis: antioxidants as mitigators. *International Journal of Molecular Sciences*.

[50] Shi Q., Liu R., Chen L. (2022). Ferroptosis inhibitor ferrostatin-1 alleviates homocysteine-induced ovarian granulosa cell injury by regulating TET activity and DNA methylation. *Molecular Medicine Reports*.

[51] Ding Y., Chen X., Liu C. (2021). Identification of a small molecule as inducer of ferroptosis and apoptosis through ubiquitination of GPX4 in triple negative breast cancer cells. *Journal of Hematology & Oncology*.

